# Wnt family member 1 (Wnt1) overexpression-induced M2 polarization of microglia alleviates inflammation-sensitized neonatal brain injuries

**DOI:** 10.1080/21655979.2022.2074767

**Published:** 2022-05-21

**Authors:** Jinzhi Gao, Hao Xu, Zhihui Rong, Ling Chen

**Affiliations:** Department of Pediatrics, Tongji Hospital, Tongji Medical College, Huazhong University of Science and Technology, Wuhan, China

**Keywords:** Microglia polarization, wnt1, LKB1, AMPK, autophagy

## Abstract

Intrauterine infection induces inflammation-mediated microglial activation and brain injury. This study aimed to explore the regulatory mechanism of Wnt family member 1 (Wnt1) in intrauterine infection-mediated microglial polarization. The cell counting kit-8 (CCK-8) assay was used to determine the viability of microglia, and cytokine expression levels were determined using enzyme linked immunosorbent assay (ELISA) kits and real-time quantitative PCR (RT-qPCR). The number of CD206^+^ and CD16/32^+^ cells was determined by flow cytometry. Wnt1 expression was analyzed using western blotting and immunofluorescence. Moreover, an *in vivo* assay was performed to verify the role of WNT1 in inflammation-sensitized brain injury in newborn mice. Lipopolysaccharide (LPS) exposure resulted in a decrease in microglial cell viability while increasing the expression levels of inflammatory cytokines (TNF-α, IL-6, and IL-1β), simultaneously promoting M1-type microglial conversion. However, these effects were rescued by overexpression of Wnt1, which was expressed less in microglia exposed to LPS *in vitro* and *in vivo*. Here, we found that Wnt1 activated the LKB1-AMPK pathway, and the inhibition of LKB1 attenuated the rescue effects of Wnt1. In addition, LPS exposure reduced the autophagy of microglia, and Wnt1 overexpression enhanced the autophagy, but this effect was reversed by treatment with an LKB1 inhibitor. Wnt1 activated LKB1 to suppress inflammation-mediated activation of microglia, promote M2-type microglia conversion via the AMPK pathway, and alleviate inflammation-sensitized neonatal brain injuries. This provides a potential avenue for the treatment of neonatal brain injuries.

## Highlights

- LPS promoted inflammation, M1-type microglia conversion and downregulation of Wnt1.
- Overexpression of Wnt1 promoted M2-type microglia conversion
- Wnt1 activated LKB1/AMPK pathway.
- Wnt1 promoted M2-type microglia conversion through the LKB1/AMPK pathway.
- Wnt1 promoted autophagy, and therefore promoted M2 polarization.

## 1. Introduction

Intrauterine infection is a common cause of cerebral palsy [1]. It increases the risk for neonatal cerebral injury and long-term neurodegeneration [2,3]. Microenvironmental changes, especially the accumulation of pro-inflammatory cytokines induced by intrauterine infection, disrupt a critical window of brain development, contributing to neuronal inflammation and the activation and M2 polarization of microglia [4,5]. Therefore, suppressing the emerging inflammatory response may be the Achilles’ heel of intrauterine infection-induced neonatal cerebral injury.

Microglia are important natural immune cells in the central nervous system and account for approximately 10% of the adult brain cells [6]. Microglia branch in the resting state and play a vital role in tissue maintenance, injury response, and pathogen defense of the central nervous system by continuously stretching and detecting the surrounding environment [7,8]. Microglia are activated in response to infection, trauma, and other stimuli in the brain and become round or amoeba-shaped, with enhanced phagocytosis and migration [9]. Activated microglia can polarize into two different phenotypes: M1 and M2 [10]. M1 has a pro-inflammatory function and plays an immune role by secreting tumor necrosis factor α (TNF-α), interleukin-1β (IL-1β), and IL-6. However, excessive inflammatory mediators, such as NO, can damage nerve cells [11,12]; Type M2 can secrete anti-inflammatory factors, such as transforming growth factor-β (TGF-β) and IL-10, to inhibit inflammation [13]. Microglial inflammation plays an important role in neonatal cerebral injury [14] and requires further study.

Autophagy is a programmed intracellular degradation process that can degrade proteins, organelles, and other substances in cells via lysosomes to maintain the metabolic balance of cells [15,16]. There are three types of autophagy: megaautophagy, microautophagy, and molecular chaperone-mediated autophagy [17]; megaautophagy is the most common type. Autophagy is beneficial for maintaining cellular homeostasis. In the case of nutrient deficiency, autophagy can protect cells and promote cell survival [18], whereas excessive autophagy can cause cell apoptosis [19]. It has been reported that autophagy is involved in regulating microglial polarization and the inflammatory response, thus affecting its survival [20,21]. In addition, autophagy mediates neuroprotective effects during brain injury [22,23]. Therefore, clarifying the relationship between autophagy, inflammation, and microglial polarization will have far-reaching significance in the study and treatment of neonatal cerebral injury induced by intrauterine infection.

Wnt protein is a secreted glycoprotein composed of approximately 350 amino acids and regulates many important links in animal development [24,25]. Wnt1 is the first member of 19 known human Wnt genes and participates in many biological processes, such as cell differentiation, proliferation, migration, and polarity formation [26]. In addition, as an extracellular growth and differentiation factor, Wnt1 is critical for nervous system development [27]. Altered Wnt1 signaling affects the metabolism of amyloid precursor proteins [28] and causes functional cognitive impairment [29]. Given the role of Wnt1 in the nervous system, this study focused on the function and regulation of Wnt1 in microglia.

Thus, the aim of this study was to explore the role of Wnt1 in neonatal brain injuries and the underlying mechanism. We hypothesized that Wnt1 regulated inflammation, microglia polarization, and autophagy via the LKB1/AMPK pathway. The study will provide a novel insight for treating neonatal brain injuries.

## 2. Materials and Methods

### 2.1 Cell culture

Mouse microglia (BV2) cells were purchased from the Type Culture Collection of the Chinese Academy of Sciences (Shanghai, China) and maintained in Dulbecco’s modified Eagle’s medium (Thermo Fisher Scientific, USA) supplemented with 10% fetal bovine serum (Gibco, Waltham, MA, USA) and penicillin/streptomycin (Gibco, Waltham). The cells were cultured in a 95%/5% (v/v) mixture of atmospheric air and CO2.

### 2.2 Cell viability assay

BV2 cells were resuspended and seeded in 96-well plates at a density of 100 μL/well. Ten microliters of cell counting kit-8 (CCK8) reagent (AmyJet Technology Co., Ltd.) was added to each well and the cells were cultured for 4 h at 37°C. A microplate reader (Nanjing DeTie Experimental Equipment Co., Ltd.) was used to measure the absorbance at 450 nm.

### 2.3 Cytokine Assay

The levels of the cytokines TNF-α, IL-6, and IL-1β in the culture supernatant were detected using ELISA kits (Beyotime, Jiangsu, China) according to the manufacturer’s instructions [30].

### 2.4 Real -time quantitative PCR (RT-qPCR)

RNA samples were extracted from all cells using a commercially available kit (Takara, Japan). Then, cDNA was synthesized, and PCR was performed using a Real-Time PCR Detection System (Bio-Rad, USA). The primer sequences used are as follows:

IL-1β: F: 5´-TGATGTTCCCATTAGACAGC-3´, R: 5'-GAGGTGCTGATGTACCAGTT-3´; IL-6: F: 5´-TCTTGGGACTGATGCTGGTG-3´,R: 5´- CAGAATTGCCATTGCACAACTC-3´; TNF-α: F: 5´-GTAGCCCACGTCGTAGCAAA-3´,R: 5´-CCCTTCTCCAGCTGGGAGAC-3´;

Wnt1: F: 5´-TACCTCCAGTCACACTCCC-3´, R: 5´-CCATGGCAGGAGAATAGGAA-3´; GAPDH: F: 5´-GAGTCCACTGGCGTCTTCAC-3´, R: 5´-ATCTTGAGGCTGTTGTCATACTTCT-3´.

### 2.5 Flow cytometry assay

BV2 cells were collected, washed twice with phosphate buffered solution (PBS), and blocked with 0.1% Triton X-100 and 3% BSA in PBS. Microglia were then stained with CD16/CD32 and CD206 antibodies (BD Biosciences). The number of microglial cells was determined using a BD FACSVerse flow cytometer (BD Biosciences).

### 2.6 Western blot

Protein extracts were subjected to 10% sodium dodecyl sulfate (SDS) gel electrophoresis. The protein extracts were then transferred to a polyvinylidene fluoride (PVDF) membrane (Millipore) and incubated with primary antibodies overnight at 4°C. The next day, the membrane was incubated with secondary antibodies at room temperature for 2 h. Finally, images were captured using an ECL system (Thermo Fisher Scientific, Inc.). The primary antibodies were anti-Wnt1 (ab15251, 1:400), anti-p-LKB1 (ab63473, 1:1000), anti-LKB1 (ab199970, 1:1000), anti-p-AMPK (ab133448, 1:2000), anti-AMPK (ab32047, 1:2000), anti-PGC1-α (ab54481, 1:1000), anti-LC3I (ab192890, 1:2000), anti-Beclin1 (ab207612, 1:2000), anti-P62(ab109012, 1:10,000) and anti-GAPDH (ab9485, 1:2500). The secondary antibody was goat anti rabbit IgG H&L (HRP) (ab205718, 1:10,000). All antibodies were obtained from Abcam.

### 2.7 GFP fluorescence microscopy

Immunofluorescence staining was performed as previous described [31]. BV2 cells were cultured in Dulbecco’s modified Eagle’s medium supplemented with 10% fetal bovine serum and then infected with GFP-tagged LC3 lentivirus (GeneChem, Shanghai, China) according to the manufacturer’s protocol. Two days later, the cells were imaged using an Olympus FluoView™ 1000 confocal microscope (Olympus, USA).

### 2.8 Intraventricular injection of Lipopolysaccharide (LPS) and transgenic mice

CX3CR1–GFP and CCR2–RFP mice were purchased from the Animal Center of the Nanjing Medical University. An intracerebroventricular injection of LPS (2 µg in P7 rats and 1 µg in P10 mice) was performed using a stereotaxic apparatus. Briefly, a 10 µL Hamilton syringe was inserted into the lateral ventricle in P7 mice with the following coordinates: 2.0 mm rostral and 1.5 mm lateral to the lambda point at a depth of 2.0 mm from the surface. For intracerebroventricular injection in P10 mice, the coordinates were 1.0 mm rostral and 1.0 mm lateral to the lambda point at a depth of 1.0 mm from the surface.

### 2.9 Statistical Analysis

Each experiment was carried out thrice. All data were analyzed using GraphPad Prism (version 7, GraphPad Software Inc.) and are presented as the mean ± standard deviation (SD). Student’s t-test was used to compare the differences between the two groups, and the contrast among multiple groups was analyzed using analysis of variance (ANOVA) followed by Duncan’s post-hoc test. The level of statistical significance was set at P < 0.05.

## 3. Results

In this study, we explore the effect of Wnt1 on neonatal brain injuries. We used RT-qPCR, ELISA, flow cytometry, and western blot to evaluate inflammation and polarization, and autophagy. The results showed that Wnt1 inhibited LPS-induced inflammation, promoted M1 to M2 conservation, and facilitated autophagy via the LKB1-AMPK pathway. The study will provide a new insight for neonatal brain injuries treatment.

### 3.1 Exposure to LPS promoted M2-to-M1 polarization of microglia

Lipopolysaccharide (LPS) was applied to culture microglia in a series of concentrations as 50,100, and 200 ng/mL. Figure 1(a) shows that the viability of microglia notably declined at concentrations of 100 and 200 ng/mL. In addition, the expression levels of IL-1β, IL-6, and TNF-α gradually increased with increasing LPS concentration (Figure 1(b,c)). Moreover, flow cytometry results showed that high concentrations of LPS resulted in a significant increase in the number of microglial cells expressing CD16/32 ^+^, while LPS did not affect the number of those expressing CD206 ^+^ (Figure 1(d-f)).

**Figure 1.** Exposure to LPS promotes M2-to-M1 polarization of microglia. (a) Cell viability of BV2 cells; (b) Levels of TNF-α, IL-6, and IL-1β in BV2 cells; (c) mRNA expression of TNF-α, IL-6, and IL-1β in BV2 cells; (d) Surface expression of CD206 and CD16/32; (e) The percentage of CD16/32 cells; (f) The percentage of CD206 cells. *P < 0.05, **P < 0.01, *** P < 0.001 versus control.

### 3.2 Wnt 1 protein expression decreased following LPS exposure

The mRNA and protein expression of Wnt1 was significantly decreased in BV2 cells and culture medium exposed to LPS (Figure 2(a-c)). Consistently, immunofluorescence results showed a similar trend: Wnt1 expression decreased in the cytoplasm of microglia exposed to LPS (Figure 2(d)).

**Figure 2.** Wnt1 protein expression decreases following LPS exposure. (a) mRNA expression of Wnt1 in BV2 cells and culture medium; (b) Protein expression of Wnt1 in BV2 cells and culture medium; (c) Quantification of (B); (d) Immunofluorescence analysis for Wnt1. *P < 0.05, **P < 0.01 versus control.

### 3.3 Wnt1 overexpression altered the polarization of microglia

To investigate the role of Wnt1 in microglial polarization, we transfected the Wnt1 overexpression vector into microglial cells and observed an increase in its expression at both mRNA and protein levels (Figure 3(a,b)). Figure 3(c) shows that Wnt1 overexpression rescued the decrease in viability of cells exposed to LPS. In addition, the expression levels of IL-1β, IL-6, and TNF-α were notably decreased with the overexpression of Wnt1 in microglia exposed to LPS (Figure 3(d,e)). Meanwhile, the number of CD16/32 ^+^ and CD206 ^+^ cells decreased and increased, respectively, after Wnt1 overexpression in microglia (Figure 3f-3h).

**Figure 3.** Wnt1 overexpression alters the polarization of microglia. (a) Expression of Wnt1 in BV2 cells and culture medium at mRNA level; (b) Expression of Wnt1 in BV2 cells and culture medium at protein level; (c) Viability of BV2 cells; (d) Levels of TNF-α, IL-6, and IL-1β in BV2 cells; (e) mRNA expression of TNF-α, IL-6, and IL-1β in BV2 cells; (f) Surface expression of CD206 and CD16/32; (g) The percentage of CD16/32 cells; (h) The percentage of CD206 cells. ##P < 0.01, ### P < 0.001 versus LPS + vector. **P < 0.01, *** P < 0.001 versus control.

### 3.4 Wnt1 suppressed LPS-induced activation of microglia

To verify the role of Wnt1 in intrauterine infections, an *in vivo* assay was performed. As shown in Figure 4(a,b), LPS injection significantly increased the number of IBA1 positive cells. However, Wnt1 overexpression significantly alleviated the effects of LPS and decreased IBA1 positive cells. Moreover, overexpression of wnt1 significantly reversed the downregulation of Wnt1 in LPS-treated mice (Figure 4(c)) and decreased the release of pro-inflammatory cytokines, such as IL-1β, IL-6, and TNF-α (Figure 4(d)).

**Figure 4.** Wnt1 alleviates LPS-induced neonatal brain injuries. (a) The expression of IBA1 was detected using an immunofluorescence assay. (b) Quantification of A. (c) The protein expression of WNT1 was determined using a western blot. (d) The release of TNF-α, IL-6, and IL-1β. **P < 0.01, *** P < 0.001.

### 3.5 Wnt1 activated the LKB1-AMPK pathway

To investigate the underlying mechanism, we measured the effect of Wnt1 on the LKB1-AMPK pathway. Western blotting was performed to analyze Wnt1, phosphorylated LKB1 (p-LKB1), LKB1, p-AMPK, AMPK, and PGC-1. The results showed that the expression of Wnt1, p-LKB1, p-AMPK, and PGC-1 was significantly decreased in cells after LPS exposure, whereas LKB1 and AMPK expression remained unchanged. Nevertheless, Wnt1 overexpression increased the expression of Wnt1, p-LKB1, p-AMPK, and PGC-1 (Figure 5(a-c)).

**Figure 5.** Wnt1 activates the LKB1-AMPK pathway. (a) Protein expression of Wnt1, p-LKB1, LKB1, p-AMPK, AMPK, and PGC1-α. (b) Quantification of p-LKB1/LKB1 and p-AMPK/AMPK ratio. (c) Quantification of each protein normalized to GAPDH. ###P < 0.001, versus LPS + vector. **P < 0.01, *** P < 0.001 versus control.

### 3.5 Wnt1 altered the polarization of microglia via the LKB1-AMPK pathway

To determine the role of the LKB1-AMPK pathway on microglial polarization, we used radicicol, an inhibitor of LKB1. The results showed that radicicol reduced the expression of Wnt1, p-LKB1, p-AMPK, and PGC-1 (Figure 6(a)). In addition, radicicol reversed the effects of Wnt1 on microglial viability after LPS exposure (Figure 6(b)). Meanwhile, the expression levels of IL-1β, IL-6, and TNF-α were notably increased after inhibition of p-LKB1 in Wnt1 overexpressing cells Figure 6(c) and Figure 5(d). In addition, the p-LKB1 inhibitor increased and decreased the number of CD16/32 + and CD206 ^+^ cells, respectively, which attenuated the impact of Wnt1 (Figure 6(e) and Figure 5(g)).

**Figure 6.** Wnt1 alters the polarization of microglia via the LKB1-AMPK pathway. (a) Protein expression of Wnt1, p-LKB1, LKB1, p-AMPK, AMPK, and PGC1-α and quantification; (b) Viability of BV2 cells; (c) Levels of TNF-α, IL-6, and IL-1β in BV2 cells; (d) mRNA expression of TNF-α, IL-6, and IL-1β in BV2 cells; (e) Surface expression of CD206 and CD16/32; (f) The percentage of CD16/32 cells; (g) The percentage of CD206 cells. &P < 0.05, &&P < 0.01, &&& P < 0.001 versus LPS + Wnt1. ##P < 0.01, ### P < 0.001 versus LPS. *** P < 0.001 versus control.

### 3.6 Wnt1 reduced the suppression of autophagy in microglia by LPS

AMPK has been reported to be a regulator of autophagy [32], and we further explored the relationship between Wnt1 and autophagy. LPS treatment significantly decreased Beclin1 and the ratio of LC3II/LC3I expression while increasing P62 expression. However, Wnt1 reversed the effects of LPS, although its action was weakened by the addition of radicicol (Figure 7a and 7b). In addition, GFP-LC3 distribution was evaluated in microglial cells, and we observed that LPS suppressed LC3 aggregation. Wnt1 promoted the aggregation of LC3, which was attenuated after LKB1 was inhibited (Figure 7c).

**Figure 7.** Wnt1 reduces the suppression of autophagy in microglia by LPS. (a) Protein expression of LC3 I, LC3 II, Beclin 1, and P62; (b) Quantification of (A); (c) GFP-tagged LC3 in BV2 cells. # P < 0.05 versus LPS + Wnt1. *** P < 0.001 versus control.

## 4. Discussion

In this study, Wnt1 overexpression suppressed the inflammatory response and promoted M2 polarization of microglia by activating the LKB1-AMPK pathway. In addition, Wnt1 overexpression alleviated LPS-induced neonatal brain injury and inhibited inflammation *in vivo*.

Microglial cells are macrophages derived from the mesoderm and are of two types, M1 and M2, after activation [33]. M2 microglia polarization is associated with numerous diseases, including cancers, inflammation, and fibrosis diseases [30,31,34]. Activated M2 microglia are involved in a series of immune responses, such as phagocytosis of apoptotic and damaged cells [35], inflammatory responses, and [36] tissue repair [37], which play a neuroprotective role. However, excessive activation of microglia to M1 type releases a large number of inflammatory factors, leading to neurotoxicity [38]. In this study, the activity of microglia treated with LPS decreased, and the release of inflammatory cytokines increased. Flow cytometry results showed that microglia were activated and converted to M1. Wnt1 inhibits microglial M1 polarization and promotes M2 polarization [39,40]. In this experiment, the expression of Wnt1 in microglia was decreased after LPS treatment, while the promoting effect of LPS on the M1-type transformation of microglia was inhibited after transferring the Wnt1 overexpression vector. Additionally, overexpression of WNT1 suppressed the inflammatory response and promoted M2 polarization, alleviating inflammation-sensitized neonatal brain injuries. These findings suggest that overexpressed WNT1 may protect against neonatal intrauterine brain injuries.

Liver kinase B1 (LKB1) is a tumor suppressor gene widely present in the human body, which encodes serine/threonine protein kinase [41] and has been reported to affect M1-M2 microglia transformation [42]. In this experiment, LPS exposure reduced LKB1 activation in microglia, whereas Wnt1 overexpression increased the activation of LKB1. To further explore the relationship between the two in microglial polarization, we used radicicol, an LKB1 activated inhibitor. The results showed that the effect of Wnt1 on microglial M2 polarization was weakened after inhibition of LKB1 activation. In addition, as an important substrate of LKB1, the AMP-actived protein kinase (AMPK) pathway plays a crucial role in neonatal brain development and injury [43]. In this study, activated AMPK and PGC1-α were both downregulated in microglia exposed to LPS, and could be rescued by Wnt1. Therefore, Wnt1 may promote microglial M2 polarization by regulating the LKB1-AMPK pathway.

It has been reported that the upregulation of autophagy promotes microglial polarization to M2 [44]. To further explore the regulatory mechanism of Wnt1 on microglial polarization, microglial autophagy was assessed, and it was found that LPS exposure could inhibit the occurrence of autophagy in microglia. After Wnt1 overexpression, the autophagy marker LC3 was reaggregated, and autophagy was promoted. However, the LKB1 inhibition weakened the action of Wnt1 in promoting autophagy.

## Conclusion

In general, Wnt1 promotes M2 polarization and autophagy of microglia by activating LKB1-AMPK signaling and alleviating intrauterine infection-induced neonatal brain injury. This may provide a potential therapeutic strategy for inflammation-sensitized brain injury in newborns.

## Supplementary Material

Supplemental Material
